# Accuracy and Cut-Off Values of Pepsinogens I, II and Gastrin 17 for Diagnosis of Gastric Fundic Atrophy: Influence of Gastritis

**DOI:** 10.1371/journal.pone.0026957

**Published:** 2011-10-31

**Authors:** Dariush Nasrollahzadeh, Karim Aghcheli, Masoud Sotoudeh, Ramin Shakeri, E. Christina Persson, Farhad Islami, Farin Kamangar, Christian C. Abnet, Paolo Boffetta, Lars Engstrand, Sanford M. Dawsey, Reza Malekzadeh, Weimin Ye

**Affiliations:** 1 Department of Medical Epidemiology and Biostatistics, Karolinska Institute, Stockholm, Sweden; 2 Digestive Disease Research Center, Tehran University of Medical Sciences, Tehran, Iran; 3 Division of Cancer Epidemiology and Genetics, National Cancer Institute, National Institutes of Health, Bethesda, Maryland, United States of America; 4 International Agency for Research on Cancer, Lyon, France; 5 Department of Public Health Analysis, School of Community Health and Policy, Morgan State University, Baltimore, Maryland, United States of America; 6 The Tisch Cancer Institute and Institute for Translational Epidemiology, Mount Sinai School of Medicine, New York, New York, United States of America; 7 International Prevention Research Institute, Lyon, France; 8 Swedish Institute for Infectious Disease Control, Stockholm, Sweden; Technische Universität München, Germany

## Abstract

**Background:**

To establish optimal cutoff values for serologic diagnosis of fundic atrophy in a high-risk area for oesophageal squamous cell carcinoma and gastric cancer with high prevalence of *Helicobacter pylori* (*H. pylori)* in Northern Iran, we performed an endoscopy-room-based validation study.

**Methods:**

We measured serum pepsinogens I (PGI) and II (PGII), gastrin 17 (G-17), and antibodies against whole *H. pylori*, or cytotoxin-associated gene A (CagA) antigen among 309 consecutive patients in two major endoscopy clinics in northeastern Iran. Updated Sydney System was used as histology gold standard. Areas under curves (AUCs), optimal cutoff and predictive values were calculated for serum biomarkers against the histology.

**Results:**

309 persons were recruited (mean age: 63.5 years old, 59.5% female). 84.5% were *H. pylori positive* and 77.5% were CagA positive. 21 fundic atrophy and 101 nonatrophic pangastritis were diagnosed. The best cutoff values in fundic atrophy assessment were calculated at PGI<56 µg/l (sensitivity: 61.9%, specificity: 94.8%) and PGI/PGII ratio<5 (sensitivity: 75.0%, specificity: 91.0%). A serum G-17<2.6 pmol/l or G-17>40 pmol/l was 81% sensitive and 73.3% specific for diagnosing fundic atrophy. At cutoff concentration of 11.8 µg/l, PGII showed 84.2% sensitivity and 45.4% specificity to distinguish nonatrophic pangastritis. Exclusion of nonatrophic pangastritis enhanced diagnostic ability of PGI/PGII ratio (from AUC = 0.66 to 0.90) but did not affect AUC of PGI. After restricting study samples to those with PGII<11.8, the sensitivity of using PGI<56 to define fundic atrophy increased to 83.3% (95%CI 51.6–97.9) and its specificity decreased to 88.8% (95%CI 80.8–94.3).

**Conclusions:**

Among endoscopy clinic patients, PGII is a sensitive marker for extension of nonatrophic gastritis toward the corpus. PGI is a stable biomarker in assessment of fundic atrophy and has similar accuracy to PGI/PGII ratio among populations with prevalent nonatrophic pangastritis.

## Introduction

Chronic atrophic gastritis is a precursor for non-cardia gastric cancer[1] and a possible risk factor for oesophageal squamous cell carcinoma (OSCC). [2] Histologic evaluation of gastric biopsy specimens is the standard way to identify atrophy, however in large epidemiologic studies measurement of serum biomarkers such as pepsinogens I, II, and gastrin-17 have been utilized as an alternative diagnostic method. [3] Pepsinogen I (PGI) is produced in the fundic glands and decreases proportionally with progression of fundic atrophy. Pepsinogen II (PGII) is synthesized in most parts of the gastric mucosa and part of the duodenum and shows no consistent pattern with fundic or antral atrophy,[4] although decrease in PGI to PGII ratio (PGI/PGII) has been shown of value for detection of fundic atrophy. [5] Gastrin is synthesized in antroduodenal G-cells and its combination with pepsinogens has been suggested as a marker for atrophy assessment [6] but the results of previous studies are not consistent on gastrin alteration with fundic atrophy.

*Helicobacter pylori(H. pylori)* infection is the key determinant in fundic atrophy development, [7] which also affects pepsinogen and gastrin secretion. [8]Patterns of *H. pylori*-induced gastritis and its outcome differ among populations. In the majority of infected individuals in developed countries inflammation is limited to the antrum with minimal involvement of the corpus and acid output remains normal or increased. [9] By contrast, in certain populations, *H*. *pylori*-induced gastritis frequently extends from the antrum to the corpus and results in pangastritis[10]which is suggested as one of the steps in progression from *H*. *pylori*-induced gastritis to fundic atrophy and gastric carcinogenesis.[11] Several cutoff values have been applied in defining fundic atrophy among different populations.[12] We hypothesize that prevalence of marked nonatrophic pangastrits in the study population might influence the accuracy and cutoff values of pepsinogens in atrophy evaluation. Eastern part of Golestan Province in Caspian littoral of Iran has some of the highest incidence rates of OSCC worldwide[13], [14], [15], [16] together with high prevalence of infection with cytotoxin-associated gene A positive(CagA+) strains of *H. pylori* (unpublished data), and high gastric cancer incidence rates. [15] The aim of the present study was to evaluate the validity of serologic diagnosis of fundic atrophy by examining the levels of PGI, PGII, PGI/PGII ratio, and G-17 against histology gold standard and also to determine influence of nonatrophic pangastritis on accuracy of serum biomarkers among patients who visited two major endoscopy clinics in the eastern Golestan province.

## Results

During study period, 329 patients aged 50 or older visited the endoscopy clinics. Dyspepsia was the main reason for performing gastroscopy. For 20 patients, blood samples were not available due to lack of consent, therefore these patients were excluded. The mean age (SD) of the included subjects was 63.5 (9.1) with a range from 50 to 90 years, and 184 (59.5%) of the participants were female.

Adequate sampling of tissue was achieved in 98% and 2% had suboptimal mass for pathological diagnosis. Oxyntic mucosa was present in 93.6% of the corpus biopsies. Fundic atrophy was observed in 21 (6.8%) patients among whom 19 also showed presence of intestinal metaplasia. In all, 101 patients were diagnosed as with nonatrophic pangastritis. In total 261 (84.5%), 22 (7.1%), and 26 (8.4%) patients were categorized as *H. pylori*+, *H. pylori*- and unknown *H. pylori* status. Kappa (95% CI) statistics for agreement between quantitative and qualitative method of *H. pylori* assessment was 0.6 (0.5–0.7). CagA+ subjects (77.5%) were significantly younger than CagA- patients (62.8 vs. 65.7 years) (p = 0.02). The CagA+ proportions among moderate and marked fundic atrophy and antral gastritis are summarized in Figure 1.

**Figure 1:** CagA+ proportion among moderate and marked fundal atrophy (dotted bar) and antral gastritis (dark bar) in comparison with no-atrophy no gastritis (diagonal lined bar) subjects.

A total of 75 subjects (24.3%) were ever tobacco users. After adjustment for histology diagnosis of fundic atrophy, there was no significant effect of age (above vs. below median)and tobacco use on PGI, PGII, PGI/PGII ratio, and G-17 levels. Male subjects were more likely to have a higher PGI level (mean difference: 26.3, 95% CI: 5.4–47.2). There were no statistical differences between men and women on the level of PGII (mean difference: 0.78, 95% CI: −3.5 −5.1) and level of gastrin (mean difference: −3.7, 95% CI: −9.9−2.5). Proportion of *H. pylori* positive was 86.4% and 87% for men and women, respectively (p = 0.89). CagA was positive among 77.6% of females and 77.2% of males (P = 0.9). The levels of PGI, PGII, PGI/PGII ratio, G-17 and *H. pylori*, CagA status are summarized in Table 1.

**Table 1:** Levels of pepsinogens, gastrin, and percentage of subjects seropositive for *H. pylori*, and CagA according to the topography of moderate/marked gastritis and atrophy.

	No gastritis No atrophy(N = 48)	Gastritis without atrophy			Gastric atrophy			P-value	
		Antral dominant (N = 74)	Corpus dominant (N = 5)	pangastritis (N = 101)	Antral (N = 60)	Corpus (N = 11)	Multifocal (N = 10)	Nonatrophic pangastritis vs. otherwise	Fundic atrophy vs. otherwise
Mean age (SD) years	63.4 (8.1)	64.2 (9.5)	63.4 (10.5)	61.5 (8.0)	65.4 (10.1)	64.5 (9.6)	66.8 (10.3)	0.45	0.27
Female/male	30/18	41/33	2/3	64/37	33/27	3/7	5/5	0.16	0.83
Current PPI use(%)	27 (56.2)	31 (41.9)	4 (80)	45 (44.5)	30 (50)	4 (36.4)	6 (60)	0.4	0.9
Mean PGI (IQR) µg/l	176.3 (108.2–241.6)	173.4 (116.9–236.8)	209 (108.7–240.1)	158.3 (118.9–245.0)	158.5 (100.9–192.8)	92.3(19.9–153.2)	72.8(18.6–126.2)	0.45	0.0001
Mean PGII (IQR) µg/l	11.3 (5.7–17.5)	13.2 (8.7–20.0)	13.9 (9.3–21.7)	17.4(12.6–28.3)	14 (11.0–20.3)	27.6(9.2–31.8)	9.7(6.0–11.5)	0.007	0.98
Mean PGI/PGII (IQR)	14.8 (10.3–17.7)	12.4 (9.6–16.3)	9.6 (9.1–11.6)	8.7 (6.9–11.2)	10.4(5.6–13.3)	3.4 (2.2–4.5)	7.8 (1.8–12.4)	0.0001	0.0001
Mean G-17 (IQR) pmol/l	10.9 (4.9–25.2)	7.1 (2.9–24.5)	33.9(18.5–82.1)	11.8 (4.9–26.9)	11.6 (5.2–21.3)	44.7(4.7–83.7)	37.5(1.4–63.3)	0.80	0.0001
*H. pylori+* (%)*	24 (50. 0)	66 (89.2)	4 (80.0)	97 (96.0)	56 (93.3)	9 (81.8)	5 (50.0)	0.0001	0.12
CagA+ (%)	23 (48.9)	49 (70.0)	4 (80.0)	91 (91.0)	54 (90.0)	7 (63.6)	6 (60.0)	0.0001	0.07

SD: Standard deviation, IQR: interquartile range, PGI: pepsinogen I, PGII: pepsinogen II, CagA: cytotoxin-associated gene A, PPI (proton pump inhibitor).

*H. pylori status was determined according to the results of histology examination, ELISA IgA/IgG, and Western blot.

The maximum J was achieved at PGI (c*)  = 56 µg/l (J = 0.55) and at PGI/PGII (c*)  =  5 (J = 0.68). Maximum J for G-17 was achieved at two points; G-17 = 2.6 pmol/l and G-17 = 40 pmol/l. Corresponding test accuracy parameters and the combinations of tests are summarized in Table 2. The proportions of PPI use and *H. pylori* infection did not differ among categories of G-17 which were produced by the G-17 cutoff points, however duration of PPI use among those with G-17>40 pmol/l was significantly longer (Table 3).

**Table 2:** Screening characteristics of PGI and PGI/PGII ratio for diagnosis of fundic atrophy and nonatrophic pangastritis.

Cutoff value	Sensitivity (95% CI)	Specificity (95% CI)	PPV	NPV	AUC (95% CI)
**Fundic atrophy**					
PGI< 56 µg/l	61.9 (38.4–81.9)	94.8 (91.6–97.1)	48.1	97.2	0.78 (0.68–0.89)
PGII > 11.8 µg/l	40.0 (19.1–63.9)	34.0 (28.6–39.8)	4.0	89.1	0.37 (0.26–0.48)
PGI/PGII< 5	75.0 (51.0–91.3)	91.0 (87.0–94.0)	35.7	98.1	0.83 (0.73–0.93)
PGI<56 and PGI/PGII<5	60.0 (36.1–80.9)	97.2 (94.6–98.8)	60.0	97.2	0.79 (0.68–0.90)
G-17<2.6 or G-17>40 pmol/l	81.0 (58.1–94.6)	73.3 (67.8–78.3)	18.1	98.1	0.77 (0.68-0-86)
PGI<56 and (G-17<2.6 or G-17>40)	57.1 (31.5–76.9)	98.6 (96.5–99.6)	75.0	96.9	0.78 (0.67–0.89)
**Nonatrophic pangastritis**					
PGI< 56 µg/l	11.5 (7.5–16.7)	97.0 (91.6–99.4)	88.9	34.8	0.54 (0.52–0.57)
PGII > 11.8 µg/l	84.2 (75.6–90.7)	45.4 (38.5–52.5)	42.9	85.5	0.65 (0.60–0.70)
PGI/PGII< 5	10.9 (5.6–18.7)	85.0 (79.4–89.6)	29.2	66.2	0.48 (0.44–0.52)
G-17<2.6 OR G-17>40 pmol/l	21.8 (14.2–31.1)	65.4 (58.5–71.8)	23.4	63.3	0.44 (0.38–0.49)

CI: confidence interval, AUC: area under curve, PPV: positive predictive value, NPV: negative predictive value, PGI: pepsinogen I, PGII: pepsinogen II, G-17: gastrin-17.

**Table 3:** Proportion of PPI use, *H. pylori* infection and fundic atrophy among categories generated by G-17 cutoff values.

		G-17 level		
	<2.6	2.6-40	>40	P-value
**Number**	39	214	55	
**Mean G-17(SD) pmol/l**	1.4 (0.6)	12.8 (9.5)	73.2(24.2)	
**PPI (%)**				
Non user	10(25.6)	39(18.3)	12(21.8)	
Former user	13(33.4)	74(34.7)	13(23.6)	0.46
Current user	16(41.0)	100(46.9)	30(54.5)	
**Median PPI use duration (IQR) (month)**				
Former users	12 (2–36)	12 (1–24)	24(12–48)	0.03
Current users	3 (0.25–36)	12 (1–24)	12 (2–24)	0.28
***H. pylori*** ** + (%)**	31(79.5.0)	190 (88.8)	47 (85.4)	0.26
**Fundic atrophy** * **(%)**	6 (15.4)	4 (1.9)	11(20)	<0.0001

G-17: gastrin-17, PPI: proton pump inhibitor, IQR: interquartile range.

*Fundic atrophy was defined by histology gold standard.

Diagnostic accuracy of PGI, PGI/PGII ratio, PGII, and G-17 to differentiate nonatrophic pangastritis and fundic atrophy are summarized in Table 2. The potentiation of PGI, PGII and G-17 in distinguishing nonatrophic pangastritis occurs independently from fundic atrophy exclusion. On the contrary, when we evaluated fundic atrophy, AUC for PGI/PGII ratio increased from 0.83 (0.73–0.93) to 0.90 (0.80–0.99) after exclusion of nonatrophic pangastritis. In assessment of nonatrophic pangastritis, receiver operating characteristic (ROC) curve revealed a differential diagnostic advantage of PGII over PGI and G-17(Figure 2). The AUC for PGII was greater than that for PGI (X^2^(1, N: 308)  = 24.9, p<0.0001) and G-17 (X^2^(1, N: 308)  = 15.1, p = 0.0001), respectively. The AUC for PGII to predict nonatrophic pangastritis was greater than that for antral gastritis (0.45 [95% CI 0.40–0.50]; X^2^ = 20.7; p<0.0001) and antral atrophy (0.49 [0.45–0.54]; X^2^ = 14.2; p = 0.0002). After restricting study samples to those with PGII<11.8, sensitivity of using PGI<56 to define fundic atrophy increased to 83.3% (95%CI 51.6–97.9) and its specificity decreased to 88.8% (95%CI 80.8–94.3).

**Figure 2:** AUCs for discrimination of fundic atrophy (dark bar), and nonatrophic pangastritis (dotted bar represents the study population after exclusion of fundic atrophy from reference group, diagonal lined bar represents whole study population). AUC: Area under curve, PGI: pepsinogen I, PGII. pepsinogen II, PGI/PGII ratio: pepsinogen I/pepsinogen II ratio, G-17: gastrin-17.

The tests for equality of the PAUCs for PGI and PGI/PGII ratio at the FPF equal to 0.05 (p = 0.95), 0.1 (p = 0.73), 0.15 (p = 0.58), and 0.20 (p = 0.56) showed no difference. The empirical PAUC for PGI and PGI/PGII ratio at FPF<0.20 was 0.06 and 0.07 respectively (p = 0.74). After dividing fundic atrophy subjects to moderate and marked, we observed an increase in AUCs (95%CI) for PGI from 0.69 (0.48–0.90) for moderate atrophy to 0.93 (0.84–1.00) for marked fundic atrophy.

Current PPI use was reported by 147(47.6%) patients with median (interquartile range) duration of 12(1–24) months. PPI use significantly increased serum levels of PGI (mean difference: 38.9, 95% CI: 19.2–58.7) and G-17 (mean difference: 6.7, 95% CI: 0.6–12.8). Exclusion of current PPI users insignificantly enhanced the sensitivity (Sen) and AUC of PGI (Sen: 81.8%, AUC: 0.88) and PGI/PGII ratio (Sen: 91%, AUC: 0.90).

## Discussion

Definitive atrophy diagnosis through endoscopy and histology examination requires invasive clinical intervention. Even histology examination that is regarded as gold standard may be subject to error due to patchy nature of atrophy and the limitation in the number of biopsies. Most of the reported specificities for serologic diagnosis of fundal atrophy are 0.9 or more. In order to calculate the optimal cut point level, we considered false positive fraction to be less than 10%.

The outcome of interest and the method of laboratory assessment vary among studies which aimed to evaluate diagnostic ability of pepsinogens. When screening of gastric cancer is purposed, PGI<70 µg/l and PGI/PGII ratio<3, measured by radioimmunoassay method, has been frequently applied as the threshold for defining population at risk in the studies from Japan.[17] Calculated cutoff values for PGI in our study was in close range with reports among dyspeptic patients in European countries[18]. Our result on similar ability of PGI/PGII ratio and PGI has been previously reported,[19] but majority of the studies showed superior ability of the joined PGI and PGI/PGII ratio[20] or the PGI/PGII ratio alone.[5], [18], [21] One explanation for this observed equal ability might be the high proportion of patients with multifocal gastritis among our study subjects. PGII has been suggested as a marker for all types of gastritis,[22], [23], and we showed that PGII behaved as a marker for nonatrophic pangastritis indifferently toward exclusion of fundic atrophy. As a result, in our population with high prevalence of pangastritis, diagnostic ability of PGI/PGII ratio was shared between fundic atrophy and multifocal gastritis which led to the attenuation of PGI/PGII accuracy in atrophy assessment. Another evidence for instability of PGI/PGII ratio over PGI came from follow-up studies on *H*. *pylori* eradication. After *H. pylori* eradication, PGI acted as a superior predictor for gastric mucosal secretion than the PGI/PGII ratio[24], partly due to the increase in PGI/PGII ratio after *H. pylori* eradication [25] which is mirrored the PGII reduction after relatively healing of inflammation. This finding suggests that PGI and PGII are markers for two different stages of fundic atrophy development. Significant change in serum PGI happens after establishment of moderate and marked fundic atrophy while PGII is sensitive to extension of inflammation toward the corpus and monitors earlier histologic changes. A recent study evaluated these markers separately and reported higher risk for gastric cancer in comparison to the ratio.[26] Several studies have looked on the association between pepsinogens and topography of gastritis [27], [28], [29], [30]. Among these studies which used PGII or PGI/PGII ratio, either absence of association [31], or presence of association with pangastritis was reported comparing with corpus-spared gastritis [32], [33], [34]. None of these studies suggested a cutoff value for PGII to distinguish pangastritis, additionally exclusion of fundal atrophy was not always among criteria of pangastritis definition. After exclusion of fundal atrophy group from pangastritis, our data suggested that PGII monitors specifically the extension of inflammation from the antrum to the corpus for the reason that its accuracy was significantly lower for corpus-spared gastritis. Because pangastritis might play a role in gastric ulcer, gastric atrophy, and gastric cancer, we further suggested a cut-off value of 11.8 µg/l with 85.5% NPV. The clinical use of this marker is limited due to its low PPV but it might be helpful to be applied in combination with other markers in multistep screening programs, however it is suggested that PGII <9.47 µg/l [35] or one fourth decrease in PGII level [36] could be used as a marker for *H. pylori* eradication. Furthermore, using PGII cutoff value in addition to PGI could help to make a more homogenous group for epidemiologic studies of atrophy association with other gastrointestinal diseases. In consistence with a study among *H. pylori* infected subjects [37] we did not observe discriminative ability of PGI, PGII, and gastrin for antral-restricted atrophy or gastritis. Despite of regulatory role of gastrin in acid secretion, in contrary with our results and an earlier study,[6] the majority of validation studies reported inadequate ability of gastrin [5], [18], [22] in fundic atrophy assessment. One explanation might be the existence of more than one cutoff point for G-17 particularly in presence of *H. pylori* infection. From our data, G-17>40 pmol/l distinguished a group of fundic atrophy in which G-cells and their negative acid-feedback remained intact and responsive to PPI, while G-17<2.6 pmol/l discriminated those atrophic stomachs with reduced antral G-cell population, damaged acid feedback, and non-responsive to PPI. However PPI use and *H*. *pylori* infection in our study sample were prevalent and contributed to hypersecretion of gastrin, thus we did not observe significant difference in their proportions among the categories with high and low cutoff values.

Compared to PGI, PGI/PGII ratio showed higher sensitivity and PPV. Because histology examination with limited number of biopsies is not a sensitive reference test, we believe this comparison is inconclusive. Low prevalence of fundic atrophy also contributed to the low PPV of the tests. Combination of G-17 and PGI increased the clinical validity in fundic atrophy assessment by improving PPV.

Similar to our results, high prevalence of *H. pylori* infection was reported by a population-based survey and a case-control study from North-western Iran [38] [39]. Additionally, using two serologic methods plus histologic examination might result in detecting higher rates of current and past *H. pylori* infection in our study. Among *H. pylori* virulence factors, CagA antigen induces longer immune response.[40] We observed a clear dose-response relationship between CagA seropositivity and severity of antral gastritis that confirmed the concept of the virulence of CagA antigen. The proportion of CagA seropositivity among fundic atrophy patients did not differ from the rest of subjects. However after excluding the marked fundic atrophy, we observed a significant higher CagA seropositivity among the fundic atrophy comparing the group without gastritis and atrophy. A similar pattern was reported in a large population-based cohort study which suggested the clearance of infection in the presence of marked fundic atrophy [41] our results supported this hypothesis.

We did not observe any elevation in pepsinogen level among male smokers. Some studies have shown that smoking increases the PGI and PGII level,[42] and other studies have reported that the association between smoking and pepsinogen disappeared when only *H. pylori* seropositive subjects were analysed.[43], [44] Due to the low number of *H. pylori* negative individuals, we were unable to assess the pepsinogen level alterations in these groups.

Absence of referral filter and high percentage of blood donation among consecutive participants are strengths of this study. One expert endoscopist performed the examination based on predesigned protocol which helped to decrease variation in biopsy localization. Also one expert pathologist reviewed the slides and it lowered the inter-observer variation for reference test. Modest sample size is one of the limitations of the study. However, it was adequate to ensure that the calculated cutoff value meets the requirement for minimum FPF. Moreover, since our study is endoscopy room-based, it is plausible that indications for endoscopy which were mostly dyspepsia symptoms, led to selection of particular group in this study. Because majority of persons with chronic gastritis or atrophy are completely asymptomatic, any generalizability toward general population should be done with caution.

In conclusion, we evaluated the accuracy of serum PGI, PGII, G-17 and CagA antibodies in assessment of fundic atrophy among endoscopy patients in an area with high prevalence of CagA+ *H. pylori* infection and upper gastroesophageal cancer. PGI<56 µg/l, PGI/PGII<5, G-17 less than 2.8 or more than 40 pmol/l were the optimal cutoff values to distinguish fundic atrophy in this population. PGI and PGI/PGII ratio showed equal accuracy in fundic atrophy diagnosis. PGI and PGII defined different steps of gastric atrophy development and establishment. PGII>11.8 µg/l was a marker for nonatrophic pangastritis, while PGI<56 µg/l distinguished the establishment of fundic atrophy insensitive to occurrence of pangastritis. The clinical use of the suggested cutoff value for PGII seems to be limited due to its low PPV but it might be helpful to be applied in combination with other markers in multistep screening programs. These findings should be replicated in studies with larger sample size and a population-based design.

## Materials and Methods

### Ethics statement

The study was approved by the ethical committee of the Digestive Disease Research Centre of Tehran University of Medical Sciences, Iran and the Stockholm Regional Ethics Vetting Board, Sweden and from all patients a written informed consent form was obtained.

### Study population

This study enrolled all dyspeptic patients over 50 years old visiting the two major endoscopy clinics of Shohada Hospital and Atrak Clinic, which are located in Gonbad city, the largest city in the eastern Golestan province, and the specialized clinics for upper gastrointestinal diseases in this area between April 2007 and August 2008 consecutively. These two clinics are the only clinics with gastroenterology specialists in eastern Golestan. The spectrum of patients varied from individuals with mild to severe gastrointestinal symptoms. Patients with a history of malignancies were excluded. Five ml of blood were taken after an overnight fast and serum aliquots were kept at −80°C. Information about tobacco, antacid, and proton pump inhibitors (PPIs) use was recorded by a trained technician during a face-to-face interview. History of PPI use during a week before endoscopy was considered as a current use. Ever consumption of tobacco regularly for at least 6 months was defined as a user.

### Histology

Endoscopies were performed by one gastroenterologist (K.A.) according to a standard protocol. Five biopsy specimens were taken from the mid-antrum greater curvature, mid-antrum posterior wall, incisura angularis, mid-corpus greater curvature, and mid-corpus posterior wall. Sections of the paraffin blocks were stained with hematoxylin and eosin (H&E) and Giemsa stains, and were submitted to the Digestive Disease Research Center laboratory for histologic examination.

All pathology slides were examined by one experienced pathologist (M.S.), using the histologic criteria of the updated Sydney System.[45] The sufficiency of each specimen for histologic examination, type of glandular mucosa, and presence of *H. pylori* were recorded. Inflammation, intestinal metaplasia, and atrophy were assessed and graded as mild, moderate or marked. Subjects with moderate or marked atrophy were combined and classified as atrophic group and those with mild or no atrophy were grouped as the non-atrophic. If one or both of the biopsies from the antrum or incisura were atrophic and the corpus biopsies were non-atrophic, the patient was diagnosed as with antral atrophy. If one or both of the biopsies from the corpus were atrophic and other biopsy sites were non-atrophic, the patient was diagnosed with fundal atrophy. When one or more biopsies from the antrum/incisura angularis and one or both biopsies from the corpus were atrophic, multifocal atrophy was mentioned as a diagnosis. The same definitions were used to describe grading and anatomic distribution of gastritis. If one or more biopsies from the corpus and at least one biopsy from the antrum/incisura angularis showed moderate or severe gastritis without atrophy, the pattern was recognized as nonatrophic pangastritis.

### Serology assays

Serum PGI, PGII and G-17 were measured, blind to histology results, using enzyme linked immunosorbent assays (ELISA) (Biohit, Finland) at the Swedish Institute for Infectious Disease Control (SMI). The coefficients of variation for PGI and PGII, using a pool of mixed serum from healthy subjects, were 7% and 14%, respectively. *H. pylori* serology was evaluated quantitatively and qualitatively, measuring cell-surface antibodies with ELISA (IgA/IgG, Biohit, Finland) and Western Blot assays (Helico Blot 2.1, MP Biomedicals Asia Pacific Ltd, Singapore), respectively. Patients were considered *H. pylori* positive if one or more of their biopsies showed presence of *H. pylori* irrespective of their serology results. They were also considered *H. pylori* positive if all of the biopsies were negative but both serology tests were positive. They were considered *H. pylori* negative when serology tests and histology results were all negative. If the results of the two serology tests were inconsistent and the histology examination was negative, the status of the patient was recorded as unknown for *H. pylori.* CagA was considered positive according to manufacturer's instructions.

### Statistical analysis

Histologic examination was used as the reference standard for diagnosing atrophy. Receiver operating characteristic (ROC) curves were constructed using different combinations of sensitivity and specificity, and the areas under the curves (AUCs) and their 95% confidence intervals (CIs) were calculated. Linear regression was used to evaluate the effects of covariates (age, gender, tobacco and current PPI use) on the levels of the pepsinogens among non-atrophic subjects. Partial AUC (PAUC) was determined at different false positive fraction (FPF) points.[46] Youden index (J) was calculated to choose the optimal cutoff value (c*) that confirmed the diagnosis of fundic atrophy or pangastritis with a FPF≤20%–30%. Stata/IC 11.0 (StataCorp LP, USA) was used for statistical calculations.
